This article has been retracted.

# Identification of Hub Genes and Immune Cell Infiltration Characteristics in Alzheimer's Disease

**DOI:** 10.1155/2021/7036194

**Published:** 2021-12-20

**Authors:** Ming Hu, Jianhua Wang

**Affiliations:** ^1^Department of Graduate School, Hebei Medical University, Shijiazhuang 050000, Hebei, China; ^2^Deparment of Neurology, Hebei General Hospital, Shijiazhuang 050051, Hebei, China

## Abstract

The purpose of this study was to identify hub genes closely correlated with Alzheimer's disease (AD) and their association with immune cell infiltration. In this work, 119 overlapping differentially expressed genes (DEGs) were obtained from GSE5281 and GSE122063 datasets through differential expression analysis. Gene Ontology (GO) and Kyoto Encyclopedia of Genes and Genomes (KEGG) pathway enrichment analyses were performed on the 119 DEGs, revealing some important biological functions and key pathways. AD immune cell infiltration analysis revealed a significant difference in the proportion of immune cells between the AD group and the control group. Finally, correlation analysis between target hub genes and immune cells indicated that GFAP had a positive or negative correlation with some specific immune cells. Our results provided useful clues, which will help to explain the molecular mechanism of AD and search for precise prognostic markers and potential therapeutic targets.

## 1. Introduction

Alzheimer's disease (AD) is a degenerative disease of the central nervous system that occurs in old age and pre-old age and is characterized by progressive cognitive dysfunction and behavioral impairment [1, 2]. It is the most common type of dementia and one of the most common chronic diseases in old age [3], accounting for about 50% to 70% of dementia in old age [4, 5]. While the exact cause of AD has not been elucidated, studies have found that AD is the result of a combination of genes, lifestyle, and environmental factors, caused in part by specific genetic changes [6–9]. A combination of drug therapy, non-drug therapy, and careful nursing can reduce symptoms and delay the progression of the disease [10–12], but there is no specific drug that can cure AD or effectively reverse the progression of the disease. The course of Alzheimer's disease is about 5–10 years, and a few patients can survive for more than 10 years. Most of them die from complications such as lung infection, urinary tract infection, and pressure ulcers [13–15]. Therefore, it is key to identify the hub genes, explore the pathogenesis, and search for the therapeutic targets of AD.

A new generation of high-throughput sequencing technologies and the development of genomics have produced a wealth of disease gene expression data and clinical information already stored in many public databases [16–18]. This provides a new idea and theoretical basis for in-depth understanding of the pathogenesis and biological characteristics of diseases through bioinformatics analysis.

In this study, we used high-throughput sequencing data for differential gene expression analysis, GO functional and KEGG pathway enrichment analyses, and protein-protein interaction (PPI) network analysis to identify network hub genes and their biological roles. In addition, we also performed immune cell infiltration analysis and correlation analysis between target hub genes and immune cells on all samples, which were main innovative points of this research paper.

## 2. Materials and Methods

### 2.1. Downloading AD Transcriptome Data from GEO Database

AD gene expression data were obtained from Gene Expression Omnibus (GEO) database [19] (https://www.ncbi.nlm.nih.gov/gds). We downloaded the GSE5281 and GSE122063 datasets using the R package GEOquery [20]. A total of 181 AD and 116 normal control samples were collected.

### 2.2. Data Cleaning and Differential Gene Expression Analysis

Firstly, the gene expression matrices of GSE5281 and GSE122063 datasets were normalized and formatted into input file format of R language. Then, the differentially expressed genes (DEGs) of AD patients were screened by robust rank aggregation [21], and the volcano plots and heatmaps of DEGs were plotted using limma [22] and pheatmap [23] packages of R. *P* value < 0.05 and | logFC (fold change) | > 1 were considered statistically significant.

### 2.3. Functional and Pathway Enrichment Analyses

To clarify the biological functions and key pathways of DEGs in AD, we performed Gene Ontology (GO), including biological process (BP), cellular component (CC), and molecular function (MF), and Kyoto Encyclopedia of Genes and Genomes (KEGG) analyses [24] using R packages such as clusterProfiler [25], enrichplot, and ggplot2 [26]. *P* value < 0.05 indicated significant differences.

### 2.4. Protein-Protein Interaction (PPI) Network Analysis

By constructing PPI networks, we could visualize the interactions between proteins, which is a powerful tool for understanding the pathological mechanisms of disease. PPI information for interesting genes was obtained from the Search Tool for the Retrieval of Interacting Genes/Protein (STRING) database (http://www.string-db.org/) [27]. Genes with a minimum required interaction score ≥0.5 were chosen to build a full network model. Then, the software Cytoscape was used to build the PPI visual network, and MCODE was used to identify the most relevant and significant modules in the PPI network [28]. Finally, the plug-in “CytoHubba” was used in Cytoscape to select the top 10 genes with the highest connectivity from the interesting genes as the hub genes of the network [29].

### 2.5. AD Immune Cell Infiltration Analysis

To compare the differences in immune cell infiltration in AD and normal tissues, we performed AD immune cell infiltration analysis by R packages ggpubr [30] and preprocessCore [31] and obtained the levels of immune cell infiltration in each sample. We then extracted the levels of immune cells in both groups (AD group and control group). The results of the differences were shown by heatmap, violin plot, and correlation matrix. *P* value <0.05 indicated statistically significant difference.

### 2.6. Correlation Analysis between Target Hub Genes and Immune Cells

To examine the association between target hub gene and immune infiltration, Pearson analysis was used to determine the correlation between gene expression and immune cell fraction by R packages limma, reshape2, ggpubr, and ggExtra [22, 31]. Firstly, the gene expression matrix and the list of immune cell infiltration results were read, and the data were collated, combined, and intersected. Then, the correlation test was calculated in cycles for all kinds of immune cells, and the correlation scatter plot was drawn. Finally, we visualized the correlation between target hub gene and immune cells with lollipop diagram.

## 3. Results

### 3.1. Identification of DEGs

Datasets GSE5281 and GSE122063 were downloaded from GEO database. The former included 87 AD brain tissue and 74 normal tissue samples, while the latter included 92 AD brain tissue and 44 normal tissue samples. After data preprocessing and gene differential expression analysis, 119 differentially expressed genes (AD/normal control tissue) were obtained using robust rank aggregation, of which 30 genes were significantly upregulated and 89 genes were downregulated in AD patients, as shown in Figures 1(a) and 1(b). The heatmap showed the top 50 DEGs with most significant upregulation and downregulation, as shown in Figure 1(c). The *P* values < 0.05 and |logFC|≥1 were the cutoff criteria.

### 3.2. GO and KEGG Enrichment Analyses of the 119 DEGs

We also ran GO function and KEGG pathway enrichment analyses for the 119 overlapping DEGs by R package clusterProfiler.  Figure 2 shows the result of GO enrichment analysis. The biological processes (BPs) of the 119 DEGs focused predominantly on chemical synaptic transmission, nervous system development, ion transport, and positive regulation of neuron projection development, as shown in Figure 2(a). With regard to the cellular components (CCs), it was found that these DEGs were strongly associated with Golgi membrane, cell junction, and neuronal cell body, as shown in Figure 2(b). Furthermore, in terms of molecular function (MF), those 119 DEGs were associated with calmodulin binding, extracellular ligand-gated channel activity, and GABA, as shown in Figure 2(c). Searching the KEGG database revealed that the DEGs mainly matched to retrograde endocannabinoid signaling, morphine addiction, and GABAergic synapse, as shown in Figure 2(d).

### 3.3. Identification of Hub Genes by PPI Network Analysis

We constructed the PPI network among these overlapping DEGs by using the STRING database and visualized them using Cytoscape software, as shown in Figure 3(a). Cytoscape was used to screen out two key modules from PPI network by MCODE algorithm, as shown in Figure 3(b). Network hub genes were identified by Degree algorithm, as shown in Figure 3(c). The top 10 network hub genes were SLC32A1, STMN2, GFAP, GABRA1, SST, GABRG2, SYN2, GNG3, PVALB, and SH3GL2, as shown in Figure 3(d).

### 3.4. Composition and Differential Expression of the Infiltrating Immune Cells

We performed CIBERSORT immune cell infiltration analysis on the GSE12206 dataset to compare the composition and differential expression of immune cells between the AD group and the normal control group.  Figure 4(a) summarizes the infiltration of 22 types of immune cells in each sample.  Figure 4(b) shows the overall composition of immune cells in AD group and control group.  Figure 4(c) shows the co-expression correlation between 22 immune cell proportions. As shown in Figure 4(d), compared with normal control group, higher proportions of T cells CD4 memory activated, macrophages M2, and neutrophils could be detected in AD group, along with lower proportions of T cells follicular helper, T cells regulatory (Tregs), NK cells activated, and mast cells resting (*P* < 0.05).

### 3.5. The Relationship between Target Hub Genes and Immune Cells

Through the PPI network analysis, we obtained 10 hub genes, among which GFAP was the upregulated gene in the AD group, so we conducted correlation analysis between GFAP and various immune-infiltrating cells. Figures 5 and 6 show the strong correlation between GFAP and immune-infiltrating cells. GFAP had a positive correlation with T cell CD4 memory activated, macrophages M2, neutrophils, plasma cells, and macrophages M1. GFAP has a negative correlation with T cells regulatory (Tregs), Mast cells resting, NK cells activated, and T cells follicular helper (Correlation Coefficient <0 and *P* value <0.05).

## 4. Discussion

AD is a central neurodegenerative disease occurring in the early and old age. It is mainly characterized by progressive cognitive dysfunction and behavioral impairment. The etiology is not clear, and there is no cure at present [32]. Therefore, it is particularly urgent to find precise prognostic biomarkers and therapeutic targets for AD. In this paper, 119 overlapping DEGs were first identified between GSE5281 and GSE122063 datasets by differential gene expression analysis. Second, GO and KEGG enrichment analyses were performed on the 119 DEGs, revealing some important biological functions and key pathways, such as chemical synaptic transmission, Golgi membrane, calmodulin binding, retrograde endocannabinoid signaling, morphine addiction, and GABAergic synapse. Also, we used the STRING database to build a PPI network among these overlapping DEGs, screened two key modules from the PPI network, and identified 10 network hub genes. They were SLC32A1, STMN2, GFAP, GABRA1, SST, GABRG2, SYN2, GNG3, PVALB, and SH3GL2. Then, we performed immune cell infiltration analysis on the GSE12206 dataset and found higher proportions of T cells CD4 memory activated, Macrophages M2, and Neutrophils in AD group, along with lower proportions of T cells follicular helper, T cells regulatory (Tregs), NK cells activated and Mast cells resting.. Finally, we analyzed the correlation between GFAP differential expression and various immune cell infiltration levels. GFAP (glial fibrillary acidic protein) is one of the groups of protein components that make up intermediate silk.

GFAP (Glial fibrillary acidic protein) is one of a group of protein components that make up intermediate silk. Intermediate filaments are found in astrocytes and help maintain normal structure and function of the brain and spinal cord. When GFAP is defective, the protein products it expresses become abnormal, which can lead to what is known as Alzheimer's diseaseh the rapid development of the automobile industry, automobile practitioners have proposed several n, a rare condition in which brain tissue is gradually destroyed. In recent years, many studies have reported the close relationship between GFAP and AD. Chatterjee et al [33]. used Simoa assay to measure plasma proteins in cognitively unimpaired older adults (CU) and found that GFAP and p-tau181 were upregulated in the CU group with cerebral amyloidosis, which indicated the clinical potential of GFAP and p-tau for the diagnosis and longitudinal monitoring of preclinical AD. Cicognola et al. [34] conducted a follow-up study of 160 patients with mild cognitive impairment (MCI) for an average of 4.7 years to detect the associated amyloid proteins in the cerebrospinal fluid. The result showed that plasma GFAP can detect the pathology of AD and predict the transformation to AD dementia in patients with MCI. Teitsdottir et al. [35] quantitatively measured novel biomarkers, including GFAP, in cerebrospinal fluid of 52 subjects using enzyme-linked immunosorbent assay (ELISA) and bioinformatics analysis. These results suggested that GFAP may be a marker of cognitive decline in predementia and early AD.

AD is a disease of the nervous system, but it also presents with systemic inflammation, with higher levels of inflammatory cytokines and chemokines in the patient's peripheral and central nerves [36, 37]. Goldeck et al. [38] studied the phenotype of circulating immune cells in AD patients by flow cytometry and confirmed that the proportion of cells expressing CD25 (a T cell CD4 memory activated) in AD patients was significantly higher than that in the control group. The proportion of CCR6+ cells was also increased, and this chemokine receptor was mainly expressed in pro-inflammatory memory cells and Th17 cells. AD patients also had a greater proportion of cells expressing CCR4 (expressed on Th2 cells) and CCR5 (Th1 cells and dendritic cells). Kasus-Jacobi et al. [39] used mass spectrometry and in vitro aggregation methods to detect the activity of neutrophil elastase (NE) and cathepsin G (CG) against amyloid-beta peptide A*β*1-42 and found that the peptide derived from CAP37 mimics the quenching and inhibitory aggregation effects of A*β*1-42 full-length protein. In addition, the peptide inhibited the neurotoxicity of the most toxic A*β*1-42 aggregates. These results provide possible strategies for the development of novel AD-modifying drugs. By constructing a neuropathic AD transgenic mouse model, St-Amour et al. [40] analyzed the important characteristics of the adaptive immune system in the serum, bone marrow, and spleen of the mice by flow cytometry and ELISPOT. The results showed that the proportion of hematopoietic stem cells decreased in the bone marrow of 12-month-old triple transgenic mouse model (3xTg-AD), and the number of lymphocytes, granulocytes, and monocytes remained unchanged. These results suggest that the 3xTg-AD model validates the adaptive immune response observed in patients with AD and confirms the activation of valuable immune pathways in AD.

Through comprehensive bioinformatics analysis, we identified the hub genes closely related to the molecular mechanism of AD, verified the biological functions and key pathways of the hub genes, and conducted immune cell infiltration analysis and correlation analysis for the target core genes. Our work will help clarify the pathogenesis of AD and provide new candidate biomarkers and potential therapeutic targets for clinical application in the future. The limitation of this study is the lack of attention to different subtypes of AD, and the results still need to be verified in vivo and in vitro.

## 5. Conclusions

In this study, we identified 10 network hub genes (SLC32A1, STMN2, GFAP, GABRA1, SST, GABRG2, SYN2, GNG3, PVALB, and SH3GL2). GFAP had a positive or negative correlation with some specific immune cells. These genes could be candidate precise prognostic markers and potential therapeutic targets.

## Figures and Tables

**Figure 1:** Identification of DEGs in the GSE5281 and GSE122063 datasets of AD. |logFC| ≥1.0 and *P* value <0.05 were set as cutoff criteria. (a) Venn diagram of DEGs between the two databases. (b) Volcano plots of DEGs in the two databases. (c) Heatmaps of the top 50 DEGs in the two databases. Red: downregulation; green: upregulation.

**Figure 2:** Bubble plots of GO and KEGG enrichment analyses of the 119 overlapping DEGs. (a) GO-BP enrichment analysis. (b) GO-CC enrichment analysis. (c) GO-MF enrichment analysis. (d) KEGG enrichment analysis. Circle size indicates the number of DEGs, and circle color indicates the *P* values.

**Figure 3:** Visualization of the PPI network and top 10 hub genes. (a) PPI network of the 54 overlapping DEGs. (b) Two key modules in the PPI network. (c) Identification of 10 hub genes from the PPI network using the Degree algorithm. Red squares: genes with high degree sores; yellow squares: genes with low degree scores. Circles or squares represent the genes or protein, and connecting lines represent interactions between them. (d) Bar chart of the top 10 hub genes.

**Figure 4:** Differences and correlation of immune cell infiltration between the AD group and control group. (a) Summary of immune infiltration in 22 immune cell subpopulations from 100 samples. (b) Heatmap of 22 immune cell infiltrations between the two groups. (c) Correlation matrix of 22 immune cell infiltration in 100 samples. (d) Violin plot of differential expression of 22 infiltrating immune cells. Abscissa: immune cell types; ordinate: relative immune cell content. Blue: AD group; red: control group.

**Figure 5:** Scatter plots of correlation in GFAP expression and different immune cell contents (a–i). (a) T cells CD4 memory activated, (b) Macrophages M2, (c) Neutrophils, (d) Plasma cells, (e) Macrophages M1, (f) T cells regulatory (Tregs), (g) Mast cells resting, (h) NK cells activated, (i) T cells follicular helper. (R) correlation coefficient; *P* < 0.05 indicates a significant correlation.

**Figure 6:** Lollipop diagram of correlation between GFAP expression and different immune cell contents. Circle size: absolute value of correlation coefficient; circle color: *P* value of correlation test. *P* < 0.05 (red) indicates a significant correlation between GFAP expression and immune cell infiltrations.

## Data Availability

The simulation experiment data used to support the findings of this study are available from the corresponding author upon request.
